# The Characterization and Functional Properties of *Euglena gracilis* Paramylon Treated with Different Methods

**DOI:** 10.1155/2022/7811014

**Published:** 2022-08-04

**Authors:** Liwei Gao, Xinjie Zhao, Xiangzhong Zhao

**Affiliations:** School of Food Sciences and Engineering, Qilu University of Technology (Shandong Academy of Sciences), Jinan 250353, China

## Abstract

*Euglena gracilis* paramylon (EGP) is a polymeric polysaccharide composed of linear *β*-1,3 glucan. The water insolubility of EGP severely limits its application. This work aimed to improve the functional characteristics of EGP by hydrogen peroxide (H_2_O_2_) degradation and carboxymethylated modification. The results showed that the crystallinity of EGP degraded by H_2_O_2_ and carboxymethylated modification decreased by 14% and 46%, and the thermal degradation temperature was significantly descending in a crystallinity-dependent manner. In addition, the results showed that H_2_O_2_ degradation and carboxymethylation significantly improved the adsorption capacity of EGP for oil, dyes, and metal ions, and their water solubility increased by 9% and 85%. This result will provide a valuable theoretical basis for the development and utilization of EGP.

## 1. Introduction

Polysaccharides are a class of molecular polymer widely existing in animals, plants, and microorganisms. Because of their safety, biocompatibility, and various biological activities, polysaccharides are commonly used in food, medicine, cosmetics, and other fields [1]. Based on the excellent biological activity and physical properties of polysaccharides, many polysaccharides have been used to improve the structural properties of food systems [2]. Nevertheless, many natural polysaccharides' weak biological activity and poor water solubility limit their broad applicability. It is worth noting that different physicochemical parameters of polysaccharides, such as monosaccharide composition, molecular structure, molecular weight, the conformation of the main chain, and branching features, play decisive roles in physicochemical properties and biological activities. Researchers have changed these polysaccharides' molecular structure and conformational characteristics to break these limitations and enhance their biological activity and physicochemical properties [3].

In recent years, the modification methods of polysaccharides include physical methods, chemical methods, and enzyme treatment methods. The enzymatic modification method is also known as the biological modification method. It has the advantages of high specificity, high efficiency, and high safety. However, it is difficult to achieve large-scale industrial production due to high cost and small number of processed samples, which seriously restricts its development. The most common physical modification methods are ultrasonication, microwave exposure, etc. The physical modification method achieves the purpose of modification by reducing the molecular weight. However, it only cuts off the original polysaccharide main chain, which has certain limitations. The chemical modification methods include sulfation [4], carboxymethylated [3], acetylation [5], and degradation [6]. The chemical methods can chemically modify the structure of polysaccharides to obtain polysaccharide derivatives with higher or new biological activities. The advantage of chemical modification is that it introduces new functional groups according to the need to change their original structure, which is more flexible than physical modification. Therefore, we choose a chemical method to modify the polysaccharides. However, most chemical modifications often have reagent residues, potentially threatening human health. Nevertheless, carboxymethylated modifications have been proven safe and nontoxic, with the advantages of simple operation and low-cost [7]. Carboxymethylated modification can change polysaccharides' structure and functional characteristics by introducing new groups to replace hydroxyl groups in polysaccharide chains. Its derivatives have potential applications in food [8]. For example, natural cellulose had no apparent biological activity and was insoluble in water, but it could be well dissolved and inhibited tumors after carboxymethylated modification [9]. Other studies have also shown that the carboxymethylated polysaccharide had more muscular biological activities such as antitumor, antioxidation, and immune regulation. Its potential mechanism is that carboxymethyl groups can effectively improve structural characteristics such as solubility and solution conformation of polysaccharides [10, 11]. H_2_O_2_ oxidation is also a common chemical degradation method of polysaccharides. It can change the biological activity of polysaccharides by dissociating to form strong oxidative hydroxyl radicals and attacking the glycosidic bond of polysaccharides. The method has the advantages of low production cost, fast degradation speed, easy industrial production, and only generates water and oxygen from the degradation, which is a green and environmentally friendly chemical degradation method. Sun et al. [6] degraded j-carrageenan with H_2_O_2_, and the results indicated that the j-carrageenan with lower molecular weights showed better antioxidant activity.

Paramylon is a storage polysaccharide from *Euglena gracilis*, a linear glucan linked by *β*-1,3 glycosidic bonds [12]. Due to the high versatility of *Euglena gracilis*, paramylon can be produced either in photoautotrophic or heterotrophic conditions, and it accumulates up to 50∼70% of the dry weight of the cell under heterotrophic growth conditions. In 2017, paramylon was approved as a novel food ingredient by the US Food and Drug Administration [13]. As one of the available active substances in *Euglena gracilis*, EGP has attracted much attention due to its various biological activities, including hepatoprotective, antiviral, and immune-stimulatory effects [14–16]. Native paramylon involves highly stable triple helices conformers, which limits the application of polysaccharides to a certain extent.

Therefore, in this study, the extracted EGP was modified by the H_2_O_2_ degradation and carboxylation method and tested by Fourier transform infrared (FTIR), scanning electron microscopy (SEM), diffraction of X-rays (XRD), and thermogravimetric (TG) analysis to explore the effect of different modifications on the functional groups' properties and internal structure of the polysaccharide. This study provides new theoretical support for expanding the development and utilization of EGP.

## 2. Materials and Methods

### 2.1. Materials and Chemicals

*Euglena gracilis* powder was purchased from the Guangyu Biological Technology Co. (Shanghai, China). Glucuronic acid, Fe^2+^, and Cd^2+^ standard solutions were purchased from Macklin Chemicals Co. (Shanghai, China). All analytical reagents were purchased from Sinopharm (Beijing, China).

### 2.2. Preparation of EGP

The *Euglena gracilis* powder was refluxed with petroleum ether (1 : 10, w/v) in an automatic Soxhlet extractor for 2 h and air-dried to obtain defatted, decolorized *Euglena gracilis* powder. Weighted a certain mass and suspended it in 10 g/L sodium dodecyl sulfate (SDS) solution, mixed evenly, took a water bath at 50°C for 1 h, centrifuged for 10 min at 6000 rpm, removed the supernatant, added 1.5 g/L SDS solution, centrifuged for 10 min at the same rotating speed, poured out the supernatant, repeated the operation twice, and finally repeatedly wash with distilled water and freeze-dried to obtain EGP [17].

### 2.3. Modified Polysaccharides

#### 2.3.1. H_2_O_2_ Degradation of Paramylon (H-EGP)

The EGP was degraded by H_2_O_2_ according to the method of Li [18] with minor modification. Dissolved the samples in a 30% H_2_O_2_ solution at a ratio of material to liquid of 1 : 5, reacted in a 40°C water bath for 3 h, centrifuged at 6000 rpm for 10 min after the reaction, and freeze-dried to obtain the H-EGP.

#### 2.3.2. Preparation of Carboxymethylated Paramylon (C-EGP)

The principle of carboxymethylated paramylon is that -OH of polysaccharide is deprotonated to form an alkoxide, and then -CH_2_COONa is introduced between chloroacetic acid and polysaccharide alkoxide [3, 7]. The solvent and water methods are often used for the carboxymethylation of polysaccharides. In this experiment, the solvent method was used to modify polysaccharides according to a previous report [19] with some modifications. Firstly, the EGP sample (1 g) was suspended in 30 mL of isopropyl alcohol. The mixture was stirred and swelled for 0.5 h with a magnetic stirrer at room temperature, followed by the addition of 30% NaOH solution to complete the alkalization process, and then 1 g of solid etherification reagent chloroacetic acid was added into the reaction bottle under stirring for 30 min. The temperature for etherification was set at 70°C and went continuously for 1.5 h to complete the etherification process. After the reaction, the precipitate after vacuum filtration was washed with absolute ethyl alcohol three times and then dried to constant weight in a 50°C oven to obtain C-EGP.

The degree of substitution (DS) could determine the degree of carboxymethyl substituted hydroxyl group, which was used to judge the success of carboxymethylation. DS is usually determined by the neutralization titration method [20]. Firstly, the C-EGP was weighed and dissolved in a 0.1 mol/L HCl solution. After sufficient shaking, the mixture was titrated with a 0.1 mol/L NaOH standard solution, and the *V*_*1*_ and *V*_*2*_ of the NaOH solution consumed at pH 2.1 and pH 4.3 were recorded, respectively. The DS could be calculated by [21]

(1) $$\begin{array}{c} DS=\frac{0.023A}{1-0.058A}, \end{array}$$

(2) $$\begin{array}{c} A=\frac{\left(V_{2}-V_{1}\right)\times C}{m}, \end{array}$$

where *V*_*1*_ is the volume of the NaOH solution consumed (mL) when pH was 2.1, *V*_*2*_ is the volume of the NaOH solution (mL) when pH was 4.3, *C* is the NaOH solution concentration (mol/L), and *m* is the mass of the EGP (mg).

### 2.4. Component Analysis of EGP and Its Modified Derivatives

The total sugar content of samples was evaluated through the calibration curve of standard glucose by the phenol-sulfuric acid method [22]. The carbazole method determined the uronic acid content, and galacturonic acid was used as the standard [23]. The rapid nitrogen determination method was used to determine the content of protein. All measurements were done 3 times.

### 2.5. Characterization

#### 2.5.1. Fourier Transform Infrared Spectroscopy

Because carboxymethyl has apparent characteristic absorption in the infrared spectrum, the FTIR can indicate whether the polysaccharide has been successfully modified. The FTIR is easy to operate and has high sensitivity, so it has been widely used to determine characteristic functional groups of polysaccharides and identify glycosidic bond configurations [4]. An FTIR spectrophotometer (Thermo Scientific, USA) was used to analyze the infrared spectrum of the samples in the range of 500 cm^−1^ to 4000 cm^−1^ with a resolution of 4 cm^−1^. The samples were mixed separately with KBr powder and ground for infrared transmission spectroscopy. Each piece was measured 3 times.

#### 2.5.2. Morphological Characteristics

According to a previous report [24], the microstructures of samples were observed using an SEM (Phenom LE, NL) of 15 kV with some modifications. The pieces were spread onto the surface of double-sided carbon adhesive tape, which was pasted onto an aluminum micrometer sheet. All samples were covered with a gold film (20 nm) in argon.

#### 2.5.3. Crystalline Characteristics

The crystallinity of EGP and its derivatives was determined using an XRD diffractometer (Rigaku Corporation, Japan) according to the description of Gui et al. [25] with minor modification: diffractograms were performed for a scattering angle of 5∼40° (2*θ*), the scanning rate was 2°/min, and a step width was set as 0.05°. The diffractograms of the samples were plotted by Origin software, and the relative crystallinity (RC,%) of the samples was calculated using the Jade 5.0 software.

#### 2.5.4. Thermogravimetric Analysis

Thermal degradation temperatures of EGP and modified derivatives were evaluated using a TG (PerkinElmer, USA). According to the method of Shibakami et al. [26] with minor modification, the experiment went on in a nitrogen atmosphere at a purge rate of 20 mL/min. Thermograms of samples (about 4.5 mg) were obtained between 30°C and 550°C at a heating rate of 20°C/min. Each group of samples was repeated 3 times.

### 2.6. Water Solubility (WS)

The water solubility of samples was determined according to the method described by Sun et al. [27] with a small modification. A dry sample (500 mg) was gently suspended with 20 mL of distilled water in a 50 mL centrifuge tube and mixed for 5 min using a vortex mixer. Prepare two copies of each sample, one in a water bath at 70°C and the other at room temperature for 20 min. The samples were centrifuged at 6000 rpm for 10 min, and the supernatant was dried at 108°C to a constant weight. The water solubility was calculated by

(3) $$\begin{array}{c} WS\left(\%\right)=\frac{m_{1}}{m_{2}}\times 10, \end{array}$$

where *m*_*1*_ is the mass of the original sample (mg) and *m*_*2*_ is the mass of supernatant after drying (mg).

### 2.7. Adsorption Capacities of EGP and Its Derivatives

#### 2.7.1. Oil Adsorption (OA) Capacity

The samples (0.5 g, dry basis) were submerged into 10 mL peanut oil and constantly stirred for 20 min at 25°C. The mixture was filtered through vacuum filtering until no oil dripped. The oil-impregnated samples were weighed. The oil adsorption capacity of samples was calculated by [28]

(4) $$\begin{array}{c} OA\left(\%\right)=\frac{w-w_{0}}{w_{0}}\times 100, \end{array}$$

where *w* is the weight of the oil-impregnated samples and *wo*  is the weight of dry samples.

#### 2.7.2. Dye Adsorption (DA) Capacity

The samples (0.2 g, dry basis) were added to 15 mL of 20 mg/L methylene blue (MB) solutions at 25°C, constantly stirring for 60 min. The dye concentration in the mixture was determined at 665 nm using a UV-Vis spectrophotometer (TU-1810, Persee, China). The methylene blue content was measured according to a standard curve. The dye adsorption capacity was calculated as follows [29]:

(5) $$\begin{array}{c} DA\left(mg/g\right)=\frac{\left(C_{0}-C_{e}\right)\times V_{0}}{m_{3}}, \end{array}$$

where *C*_*0*_ and *C*_*e*_ are the dye concentration in the solution before and after adsorption, respectively, *V*_*0*_ is the volume of the dye solution, and *m*_*3*_ is the weight of the samples.

#### 2.7.3. Metal Ion Adsorption (MIA) Capacity

The samples (0.2 g, dry basis) were submerged into the 10 mg/L metal ion solution (Fe^2+^, Cd^2+^) at room temperature, agitating continuously for 12 h. After carbonization and ashing, the immersed samples were used to measure the concentration of metal ions in the solution at specific wavelengths by an atomic absorption spectrometer (PinAAcle 900Z, PerkinElmer, USA). The metal ion concentration was determined according to a standard curve. The adsorption capacity of metal ion was calculated as follows [30]:

(6) $$\begin{array}{c} MIA\left(mg/g\right)=\frac{\left(C_{1}-C_{2}\right)\times V_{e}}{m_{4}}, \end{array}$$

where *C*_*1*_ and *C*_*2*_ are the concentrations of metal ions before and after adsorption, respectively, *m*_*4*_ is the weight of the samples, and *V*_*e*_ is the volume of the metal ion solution.

### 2.8. Statistical Analysis

All the data were shown as means ± standard deviations (SD) of three replicated determine. Statistical analysis was performed with the analysis of variance (ANOVA) using IBM SPSS Statistics software.

## 3. Results and Discussion

### 3.1. Chemical Analysis and DS

The total sugar, uronic acid, protein content, and DS of the three samples are summarized in Table 1. The results showed that samples had undergone significant alterations in chemical composition after using different modification methods. The total sugar contents of the samples were 55.06% (EGP), 48.39% (H-EGP), and 44.73% (C-EGP), showing a specific downward trend. In addition, the protein contents of the three samples were less than 1%, indicating that protein was removed effectively. The DS of C-EGP was 0.14, which demonstrated that carboxymethylation was successful. Compared with EGP, the uronic acid content (23.59%) was increased after carboxymethylation treatment; the difference between C-EGP and EGP could be due to the *β*-elimination reaction of the carboxymethylation period in alkaline conditions [31]. A previous study reported that the addition of sulfate and carboxymethyl functional groups decreased total sugar content [27]. In another study, the protein content was relatively reduced, while the entire sugar content and uronic acid of modified corn silk polysaccharides were increased significantly [32]. It could be seen that different modification methods could change the chemical composition of polysaccharides, but the results were not consistent.

### 3.2. FTIR Spectroscopy Analysis

After successful carboxymethylation, the -OH groups of the polysaccharide chain were replaced by carboxymethyl groups, leading to the changes in configuration and conformations of the main chain of the polysaccharide and the physicochemical properties [33]. FTIR can determine the position of the carboxymethyl substituent according to the characteristic absorption of carboxymethyl groups in the spectrum. For example, the carboxymethylated polysaccharide from *Morchella angusticepes Peck* showed two new peaks at 1424 cm^−1^ and 1330 cm^−1^ in the infrared spectrum, indicating carboxymethyl groups were successfully introduced [34].

Figure 1 shows the infrared spectra analysis of EGP and its modification products. A massive peak at 3354 cm^−1^ (O–H stretching vibration) illustrated that these samples contain characteristic absorption peaks of polysaccharides. The height around 2900 cm^−1^ was C-H trying in CH_2_ and CH_3_ radicals, 1036 cm^−1^ was the ether ring (C-O-C) stretching vibration peak on the sugar ring, and 887 cm^−1^ was the *β*-glycosidic bond absorption peak. It could be seen from the spectra that the infrared range of EGP was consistent before and after modification with hydrogen peroxide, indicating that the functional groups of EGP did not change after oxidative degradation. The characteristic absorption peaks of carboxymethylated polysaccharides are related to stretching vibrations of C=O groups. The absorption peaks of C-EGP at 1595 cm^−1^ and 1319 cm^−1^ were assigned to the stretching vibrations of -COO. In addition, other absorption peaks have also revealed the changes in polysaccharide structure by modification. For example, the characteristic absorption peaks of carboxymethylated polysaccharides are also related to stretching vibrations of C=C groups [35]. The peak at 1413 cm^−1^ was C-C vibrations, proving that C-EGP has been successfully carboxymethylated.

### 3.3. Surface Morphology Analysis

SEM observed the morphological changes of the EGP before and after H_2_O_2_ degradation and carboxymethylation modification. The size and shape of the surface of EGP, H-EGP, and C-EGP were significantly different in the SEM images. The EGP was oval with a uniform and smooth surface (Figure 2(a)). The surface of H-EGP was cracked to varying degrees, and even the shape of the sample changed (Figure 2(b)). Compared with the H-EGP, the C-EGP had a more significant change in structure. The C-EGP was broken into fragments, and its surface roughness was significantly increased (Figure 2(c)). Ma et al. [36] found the morphology of *Inonotus obliquus* polysaccharide showed pieces without uniform sizes, with particles similar to tiles after carboxymethylation modification. Besides, other research also found that polysaccharides showed irregular fragments after carboxymethylation treatment, while polysaccharides before treatment had a smooth appearance of different sizes [3, 37].

### 3.4. XRD Analysis

The XRD spectra of the samples are indicated in Figure 3. EGP had a sharp and narrow peak at 7°, 19°, 21°, and 24°, and three small peaks at 12°, 14°, and 17° (Figure 3(a)). After H_2_O_2_ treatment, the crystallization areas of EGP hardly changed. After carboxymethylation treatment, the XRD images of EGP changed, the peak heights of crystal peaks at 7°, 19°, 21°, and 24° decreased obviously, and three small peaks at 12°, 14°, and 17° disappeared. Figure 3 shows that the crystallinity of H-EGP and C-EGP decreased compared with EGP, which meant that the initially ordered arrangement of EGP was disturbed.

### 3.5. Thermogravimetric Analysis

Thermogravimetric analysis (TG) and differential thermogravimetric (DTG) curves are shown in Figure 4. The weight losses and degradation temperatures of EGP and its derivatives are presented in Table 2. In all samples, the DTG curves showed two steps of weight loss. The initial weight loss stage in the range of 30∼150°C was usually attributed to the loss of water [38]. At 150∼550°C, the second stage of weightlessness was related to the destruction of hydrogen bonds and the decomposition of EGP [39]. The degradation temperature of H-EGP was lower than EGP (266.17°C), which may be due to the degradation of the modified substance and the increase in the crack surface area. The degradation temperature of C-EGP decreased from 266.17°C to 188.65°C, which may be due to the destruction of the crystallization zone after modification.

### 3.6. Water Solubility and Adsorption Capacity Analysis

Polysaccharides are usually insoluble in water due to their high molecular weight, limiting their application in some fields. Good water solubility is significant for polysaccharides to exert their functional properties [40].

Carboxymethylated modification can improve the solubility of polysaccharides in water. For example, the water solubility of *Ganoderma lucidum* polysaccharide was significantly enhanced by carboxymethylated [36]. The water solubility test found that EGP was dispersed in water at 25°C or 70°C, which was closely related to its high molecular weight and crystallinity [15]. The solubility of H-EGP was 2.45% at 25°C, which may be related to the degradation of polysaccharides. It could be seen from the experimental data in Table 3 that the water solubility of C-EGP at 25°C was close to the water solubility at 70°C, and the water solubility of C-EGP was increased by 79.67% compared with EGP. Carboxymethyl groups have excellent hydrophilicity, and the hydrogen bonds between carboxymethyl groups and water increase with the increase of the number of carboxymethyl groups, which can reduce the formation of intramolecular hydrogen bonds and significantly improve the solubility [10].

The samples' adsorption capacity of oil, dye, and metal ions is listed in Table 3. The results showed that modification significantly improved the adsorption capacity of EGP. Compared with EGP, the oil absorption of H-EGP and C-EGP increased by 1.3 times and 2 times. Similarly, the adsorption capacity of H-EGP and C-EGP for methylene blue (MB) increased by about 1.4 times and 2 times. These data showed that C-EGP adsorbed more oil and MB. It was speculated that carboxymethylated modification might provide a larger amorphous region, which increased the adsorption capacity [41]. In addition, the adsorption capacities of H-EGP for Fe^2+^ and Cd^2+^ were 0.15 mg/g and 0.16 mg/g, respectively, while the adsorption capacities of C-EGP for Fe^2+^ and Cd^2+^ were 0.23 mg/g and 0.22 mg/g. Although both modification methods enhanced the adsorption capacity of EGP, the adsorption principle was different. The improvement in the adsorption capacity of H-EGP was due to the increase in the specific surface area. But for C-EGP, it was more inclined to introduce carboxymethyl groups, and C-EGP′ electron cloud density and electron-withdrawing activity increased, thereby increasing the interactions with metal ions [42].

## 4. Conclusions

The structural modification of polysaccharides can affect their functional properties and biological activities. This study examined the effects of H_2_O_2_ degradation and carboxymethylated modification of EGP on the structural and functional properties. The chemical composition of EGP was changed after two kinds of modifications. The FTIR proved that the structure of EGP did not change after H_2_O_2_ degradation, and the infrared spectrum of C-EGP showed a new characteristic absorption peak, which indicated that the carboxymethyl group was successfully introduced. The microstructural analysis indicated that the H-EGP particles appeared to have cracks; however, EGP particles were broken, and the surface became rough after carboxymethylation modification. In addition, the crystalline region and thermal stability of H-EGP and C-EGP were reduced, but C-EGP was more obvious. Through the water solubility test, we found that the solubility of the modified polysaccharide has been significantly improved, which would further expand the application of polysaccharides in food, medicine, and other industries. It was worth noting that the EGP's adsorption capacity for oil, dye, and metal ions was increased about 2 times after carboxymethylated treatment, and the C-EGP was expected to appear as a new green absorbency.

## Figures and Tables

**Figure 1:** FTIR spectra of EGP and its derivatives.

**Figure 2:** SEM images of samples. (A-1, A-2) EGP, (B-1, B-2) H-EGP, and (C-1, C-2) C-EGP.

**Figure 3:** XRD diffraction diagrams of EGP and its derivatives. (a) EGP, (b) H-EGP, and (c) C-EGP.

**Figure 4:** TG (a) and DTG (b) curves of EGP and its derivatives.

**Table 1:** Chemical composition of EGP, H-EGP, and C-EGP.

Samples	EGP	H-EGP	C-EGP
Total sugar (%)	55.06 ± 0.992^a^	48.39 ± 0.456^b^	44.73 ± 0.300^c^
Uronic acid (%)	19.76 ± 1.348^b^	22.34 ± 0.187^a^	23.59 ± 0.374^a^
Protein (%)	0.74 ± 0.045^a^	0.68 ± 0.066^a^	0.53 ± 0.045^b^
DS	/	/	0.14 ± 0.031

Values are mean ± SD, *n* = 3. Values in the same column with different letters are significantly different (*p* < 0.05).

**Table 2:** Thermogravimetric analysis of the EGP and its derivatives.

Sample	First-stage weight loss (30∼150°C)		Second-stage weight loss (150∼550°C)		Residue (%)
	T_d1_ (°C)	Δw_1_ (%)	T_d2_ (°C)	Δw_2_ (%)	
EGP	57.38 ± 0.382^a^	2.26 ± 0.248^c^	266.17 ± 1.071^a^	82.46 ± 0.649^a^	14.44 ± 1.065^b^
H-EGP	34.63 ± 0.601^b^	12.95 ± 0.567^a^	258.54 ± 1.319^b^	72.88 ± 1.215^b^	14.01 ± 0.235^b^
C-EGP	56.66 ± 0.642^a^	3.00 ± 0.155^b^	188.65 ± 0.768^c^	25.19 ± 0.306^c^	70.63 ± 1.036^a^

Data are expressed as means ± SD (*n* = 3).

**Table 3:** Adsorptive capacity and water solubility of EGP and modified derivatives.

Sample	Adsorptive capacity			Water solubility		
	Oil (g/g)	MB (mg/g)	Fe^2+^ (mg/g)	Cd^2+^ (mg/g)	25°C (%)	70°C (%)
EGP	0.30 ± 0.036^b^	0.34 ± 0.021^c^	0.04 ± 0.026^c^	0.11 ± 0.025^c^	0.52 ± 0.271^c^	0.60 ± 0.157^c^
H-EGP	0.40 ± 0.057^b^	0.46 ± 0.031^b^	0.15 ± 0.025^b^	0.16 ± 0.015^b^	3.31 ± 1.033^b^	8.89 ± 2.338^b^
C-EGP	0.61 ± 0.060^a^	0.70 ± 0.051^a^	0.23 ± 0.015^a^	0.22 ± 0.015^a^	80.19 ± 2.096^a^	85.10 ± 2.612^a^

Data are the mean ± SD of a triplicate analysis. Values in the same column with different letters were significantly different at the 5% level.

## Data Availability

The data used to support the findings of this study are included within the article.
